This article has been retracted.

# Inhibition of Oxidative Stress: An Important Molecular Mechanism of Chinese Herbal Medicine (Astragalus membranaceus, Carthamus tinctorius L., Radix Salvia Miltiorrhizae, etc.) in the Treatment of Ischemic Stroke by Regulating the Antioxidant System

**DOI:** 10.1155/2022/1425369

**Published:** 2022-05-23

**Authors:** Xixi Zhao, Yu He, Yangyang Zhang, Haofang Wan, Haitong Wan, Jiehong Yang

**Affiliations:** ^1^School of Basic Medical Sciences, Zhejiang Chinese Medical University, Hangzhou 310053, China; ^2^School of Pharmaceutical Sciences, Zhejiang Chinese Medical University, Hangzhou 310053, China; ^3^Academy of Chinese Medical Sciences, Zhejiang Chinese Medical University, Hangzhou 310053, China; ^4^School of Life Sciences, Zhejiang Chinese Medical University, Hangzhou 310053, China

## Abstract

Ischemic stroke is a severe cerebrovascular disease with high mortality and morbidity. Traditional Chinese medicine (TCM) has been utilized for thousands of years in China and is becoming increasingly popular all over the world, especially for the treatments of ischemic stroke. More and more evidences have implicated that oxidative stress has been closely related with ischemic stroke. This review will concentrate on the evidence of the action mechanism of Chinese herbal medicine and its active ingredient in preventing ischemic stroke by modulating redox signaling and oxidative stress pathways and providing references for clinical treatment and scientific research applications.

## 1. Introduction

Cerebrovascular disease is a common neurological disease, which refers to brain dysfunction caused by various vascular diseases [1]. Stroke is the main clinical type of cerebrovascular disease. Among them, atherosclerosis has been well-recognized as one of the main culprits for the rising incidence of stroke-related mortality [2]. Plaque rupture and thrombosis result in the acute clinical complications of stroke. Ischemic stroke accounts for most cases (87%) in stroke and is further subtyped into atherosclerosis, cardioembolic, lacunar, other causes, and cryptogenic strokes [3]. Therefore, atherosclerosis is an important cause of ischemic stroke [4].

Ischemia/reperfusion (I/R) injury refers to a condition in which tissues or organs suffer from ischemia for a period of time and then supplement with oxygen-enriched blood (reperfusion), resulting in aggravated tissue or organ damage. Reperfusion is essential for protecting the injured brain tissue, but it can also lead to reperfusion injury by exacerbating the damage despite restoring the circulation [5]. Cerebral I/R injury further aggravates the pathological damage of cerebral ischemic tissue and the nervous system and even produces irreversible nerve damage and clinical symptoms [6]. Cerebral I/R injury is a very complex cascade of pathophysiological processes involving multiple pathogenic mechanisms, including inflammation, oxidative stress, Ca^2+^ overload, excitatory amino acid toxicity, and mitochondrial damage, which ultimately lead to neuronal necrosis and apoptosis [7, 8]. Among them, oxidative stress is one of the important pathological mechanisms of the occurrence and development of cerebral I/R injury.

With the continuous deepening of relevant basic research, further exploration of the pathogenesis of ischemic stroke and finding effective drugs are the focus of the current research. Studies have shown that traditional Chinese medicine (TCM) has ameliorating effects on cerebral microcirculation disorders, cerebral damage, and neuronal damage caused by ischemic stroke [9].

In this review, we will first discuss the redox signaling and oxidative stress pathways in ischemic stroke. Simultaneously, we summarize the antioxidant effects of some Chinese herbal medicines, which have inhibition effects on ROS generation and oxidative stress after ischemic stroke. And we have provided a reference basis for clinical treatment and scientific research application.

## 2. Oxidative Stress and ROS

Oxidative stress is defined as an imbalance between the production of free radicals and the capacity of the antioxidant defense system [10]. This imbalance leads to damage of important biomolecules and organs with potential impact on the whole organism. It is also considered as a critical component of the pathogenesis and progression of brain disease, such as stroke and Alzheimer's and Parkinson's diseases [4, 11–13]. Free radicals can be divided into two categories: reactive oxygen species (ROS) and reactive nitrogen species (RNS). ROS and RNS are well recognized for playing a dual role as both deleterious and beneficial species, since they can be either harmful or beneficial to living systems. Enzymatic antioxidant defenses include superoxide dismutase (SOD), glutathione peroxidase (GSH-Px), and catalase (CAT); nonenzymatic antioxidants are represented by ascorbic acid (vitamin C), *α*-tocopherol (vitamin E), glutathione, carotenoids, flavonoids, and other antioxidants [14]. Under normal conditions, the free radicals produced by the human body can be eliminated in time by the antioxidant enzymes in the body, so that the generation and elimination of free radicals are in a dynamic balance. This balance is essential for the survival of organisms and their health. When the content of ROS plus RNS in the body exceeds the scavenging ability of its own antioxidant defense system, it can destroy the original redox homeostasis, trigger a variety of damage mechanisms to destroy the antioxidant defense system, and produce oxidative stress [15].

ROS are products of a normal cellular metabolism, including superoxide anion, hydrogen peroxide (H_2_O_2_), hydroxyl radicals, and singlet oxygen. Most ROS are generated by the mitochondrial respiratory chain in cells [16]. In addition, ROS is also produced by a variety of enzymes, such as NADPH oxidase (NOX), xanthine oxidase, nitric oxide synthase, and other zymogen systems [16]. ROS plays an important role in both physiological and pathological processes. Beneficial effects of ROS occur at low/moderate concentrations and involve physiological roles in cellular responses to anoxia, as for example in the function of a number of cellular signaling systems [17]. But when they are overproduced, it will cause energy depletion and accumulation of toxic substances in the cell, which will eventually lead to cell necrosis [18]. ROS produced during the ischemia and perfusion phases of acute ischemic stroke can lead to brain damage [19].

## 3. Antioxidative Systems Related to Ischemic Stroke

The state of oxidative stress produced by the destruction of the homeostasis between the body's oxidation and antioxidant systems is the key mechanism underlying ischemic stroke [20]. Oxidative stress can cause inflammation, neuronal apoptosis, excitotoxicity, and damage to the blood-brain barrier, which can aggravate brain damage [21, 22]. Therefore, it is very important to regulate oxidative stress on the biological effects of ischemic stroke and its pathogenesis. Thioredoxin (Trx), glutathione (GSH), and nuclear factor erythroid 2-related factor 2 (Nrf2) systems are three major antioxidant systems responsible for removing overproduced free radicals (Figure 1).

### 3.1. Nrf2 System

Nrf2, as a key component of endogenous antioxidant defense, and a key transcription factor that maintains cell redox homeostasis, has been demonstrated to protect the brain against stroke-induced injury mostly by alleviating ROS-associated pathological processes [23].

Under basal conditions, Nrf2 is sequestered by cytoplasmic kelch-like ECH associated protein 1 (Keap1) and targeted to proteasomal degradation [24]. Under oxidative stress, Nrf2 dissociates from Keap1 and transfers to the nucleus to promote the transcription of antioxidant response element- (ARE-) dependent genes [25]. These stress conditions lead to the suspension of Keap1–Nrf2 interactions and promote the transcription of a wide variety of antioxidant genes like heme oxygenase-1 (HO-1) and NAD(P)H:quinone oxidoreductase 1 (NQO1), which, in turn, scavenges the cellular oxidative stress [26].

*In vivo* study has shown that in both peri-infarct and core infarct regions, Nrf2 expression began to increase at 2 h, peaked at 8 h, then decreased at 24 and 72 h of reperfusion in a mouse transient middle cerebral artery occlusion (tMCAO) model [27]. At the same time, it was found that after 24 h of reperfusion, the Nrf2 signaling pathway was obviously activated after drug intervention; the levels of SOD, CAT, Nrf2, HO-1, and NQO-1 increased; and the levels of MDA, 4-hydroxynonenal (4-HNE), 8-hydroxy-2′-deoxyguanosine (8-OHdG), and ROS decreased, in a rat MCAO model [28]. And knockdown of Nrf2 abolished the protective effects of drugs on cell viability and reversed the downregulation of Nrf2 downstream gene levels induced by drugs [28]. In summary, the Nrf2 system plays an important role in regulating the redox steady state.

### 3.2. GSH System

GSH system comprises NADPH, glutathione reductase (GR), and GSH. GSH is an important nonenzymatic endogenous antioxidant in the human body and is a major endogenous component of the cellular antioxidant defense [29]. It is capable of scavenging various ROS directly to provide protection from oxidative stress-induced damage. GSH is produced intracellularly from three amino acids—glutamate, cysteine, and glycine—through two consecutive steps catalyzed by *γ*-glutamyl cysteine ligase (GCL, also known as *γ*-glutamyl cysteine synthetase) and GSH synthetase (GS) [30]. In the redox reaction, GSH is oxidized and converted into glutathione disulfide (GSSG), which is subsequently reduced to GSH by glutathione reductase [31]. Reduced form glutathione plays key roles in the cellular control of ROS. Thus, the ratio of GSH/GSSG is a good measure of the oxidative stress of an organism [32].

It is reported that the active form of GSH is most abundant in neurons and myelinated axons in a variety of brain regions including hippocampal CA1 neurons, frontal cortex pyramidal neurons, and reticular formation neurons in the unperturbed adult mouse brain [33]. The reduced form of GSH is constitutively synthesized in neurons and readily diffuses into the nucleus to protect DNA from oxidative damage [33]. Researchers found that the GSH levels in mouse CA1 pyramidal neurons were decreased during the first few hours of I/R, accompanied by increased superoxide levels; conversely, the prevention of ischemia/reperfusion-induced increase in superoxide production using an inhibitor of nicotinamide adenine dinucleotide 3-phosphate oxidase, a major source of ROS, was found to suppress the decline in GSH in postischemic neurons [34]. Another literature demonstrated that GSH reduces the brain infarct volume after MCAO injury in the rat brain and attenuates the production of ROS in brain endothelial cells after ischemic injury [35].

These data suggest that abatement of GSH can help reduce the oxidative stress response after I/R injury and relieve the severe brain lesions caused by ischemic stroke. In summary, GSH also plays a vital role in regulating the body's redox homeostasis.

### 3.3. Trx System

Trx system consists of two types of antioxidant oxidoreductase proteins: Trx and thioredoxin reductase (TrxR) and NADPH as the electron donor [36]. This system operates by transferring electrons from NADPH via TrxR to the active site of Trx [37]. It is widely present in prokaryotic and eukaryotic organisms [38]. Trx is a 12 kDa protein ubiquitously expressed in all living cells, characterized by the highly conserved reduction/oxidation- (redox-) active site sequence Trp-Cys-Gly-Pro-Cys-Lys [39]. The two cysteine residues within the redox-active center of Trx (Cys-32 and Cys-35) are the key for it to regulate redox [37].

Mammalian cells contain two distinct Trxs. Trx1 is localized in the cell cytosol/nucleus, whereas Trx2 is a mitochondrial protein [40]. One literature reported that intracellular Trx1 overexpression has a neuroprotective effect during short duration ischemia and reperfusion [41]. Ischemic neuronal death was attenuated, and superoxide production was decreased after mild focal ischemia in Trx1 transgenic mice [41]. Researchers applied RNA interference targeting Trx1 in a rat model of MCAO-induced focal ischemia. They found that administration of Trx1 siRNA significantly increased mortality, brain infarct size, neurobehavioral deficits, and neuronal cell death in MCAO rat [42]. And in the ischemic brain, administration of antioxidant enzymes peroxiredoxin 3 and Trx2 shows substantial neuroprotective effects by reducing oxidative stress [43].

These data suggest that abatement of Trx may be harmful in cerebral ischemia in the acute phase, and an elevation of Trx could be neuroprotective with respect to brain damage. In short, the Trx system can play a protective role through antioxidant effects to reduce neuronal damage caused by ischemic stroke.

## 4. Protective Effects of TCM and Its Constituent Compounds on Ischemic Stroke

### 4.1. Ligusticum chuanxiong

*Ligusticum chuanxiong* (LC), a crude herbal drug isolated from the dried root or rhizome of *Rhizoma Chuanxiong*, has been widely used in the treatment of brain and heart diseases. Pharmacological investigations demonstrate that LC possesses antiatherosclerosis, anticancer, antioxidant, antiaging, and antihypertensive properties [44]. Some researchers found that the main active ingredients in LC alcohol extract are ligustrazine, ferulic acid, free phenol, and bound phenol. After the LC alcohol extract is diluted 100 times, the reducing power was equivalent to14.79 *μ*g/mL VC. The clearance rate of 0.9 g/L LC alcohol extract on hydroxy radical was 1.12 times that on superoxide anion, which means the LC alcohol extract has a better scavenging effect on hydroxyl free radicals than superoxide anion [45]. Ligustrazine, also called tetramethylpyrazine, is a main active fraction of the traditional medicine known as LC, which has been proven to regulate the production of oxidative stress and ROS, and is used as clinical medication for cerebral thrombosis, coronary heart disease, and stenocardia recently [46]. Ligustrazine 20 mg/kg increased Nrf2/HO-1 signaling in neutrophils after ischemia [47]. The volatile oil from Chuanxiong can promote the life of cerebral cortex neurons in vitro; decrease cerebral infarction volume; enhance the activities of SOD, GSH-Px, and nitric oxide synthase(NOS); decrease the content of MDA in rats; and alleviate the damages caused by ischemia reperfusion [48].

### 4.2. Astragalus membranaceus

*Astragalus membranaceus* was first recorded in the *Shennong Bencao Jing*, one of the most famous Chinese ancient books in 200 AD, which is nontoxic and has a wide range of therapeutic effects [49, 50]. In China, it is known as “Huangqi.” It is used to invigorate the spleen and replenish qi in TCM. Huangqi abounds with polysaccharides, flavonoids, saponins, amino acids, and other compounds [51, 52].

Early literature reported that total flavonoids of *Astragalus membranaceus* had potent antioxidant activity to improve atherosclerosis [53]. As one of the fundamental components in the root of *Astragalus membranaceus*, astragaloside IV (AST IV) exerts protective effects against neurological disorders, such as cerebral I/R injury [54, 55]. Studies have found that AST IV treatment could obviously increase SOD and LDH activities; reduce the production of NOS, MDA, and NO; and downregulate the expression of inducible nitric oxide synthase (iNOS) mRNA to ameliorate the oxidative damage in rats with cerebral I/R injury [56]. What is more, it could alleviate cerebral I/R injury through inhibiting NLRP3 inflammasome-mediated pyroptosis via activating Nrf2 [57]. Meantime, AST IV-tetramethylpyrazine played a pivotal synergistic protective role against focal cerebral ischemic reperfusion damage in a rat experimental model, which could downregulate MDA content and iNOS activity, and upregulate SOD activity [58]. *Astragalus polysaccharides* (APS) are the main active ingredient of *Astragalus membranaceus*, which could also reduce NOS, LDH, NO, and MDA and increase the activities of SOD in the cerebral I/R injury model [59]. Calycosin-7-*O*-*β*-*D*-glucoside is also a representative isoflavone isolated from the root of *Astragalus membranaceus*, which has potential neuroprotective effects [60]. In vitro pharmacological studies indicated that it could alleviate oxygen-glucose deprivation/reoxygenation- (OGD/R-) induced oxidative stress in hippocampal cells by reducing the production of ROS and MDA [61].

### 4.3. Radix Salvia Miltiorrhizae

*Radix Salvia Miltiorrhizae*, as known as “Danshen,” a famous Chinese herb medicine, has been widely used in treating stroke. The active ingredients in Danshen are mainly divided into fat-soluble tanshinone compounds and water-soluble salvianolic acids [62]. The water-soluble salvianolic acids include salvianolic acid A, salvianolic acid B, salvianolic acid C, protocatechuic acid, danshensu, and other derivatives [63]. The fat-soluble tanshinone compounds include tanshinone I, tanshinone IIA, dihydrotanshinone, isotanshinone IIA, and isocryptotanshinone [62]. Both of them have significant pharmacological activities, such as antioxidant and anti-inflammatory [63–65]. Salvianolic acid B is the main active ingredient of Danshen, which could increase the level of antioxidant substances and decrease free radicals' production [66]. Experimental studies have shown that salvianolic acid B can significantly raise the activities of SOD, CAT, GSH-Px, and total antioxidant capacity (T-AOC) and reduce the levels of MDA, LDH, and NOS in cerebral ischemia model animals [66, 67]. Danshen polysaccharide is a kind of polysaccharide extracted from the root of Danshen. One literature reported that pretreatment with Danshen polysaccharide for 10 days prior to the blocking bilateral common carotid artery occlusion also significantly increased mitochondria SOD, CAT, and GSH-Px activities and reduced MDA production in cerebral ischemia brain [68]. And tanshinone IIA elicits a neuroprotective effect through attenuating oxidative productions, increasing antioxidant enzyme activity and Nrf2 expression, and inducing Nrf2 nuclear translocation [69].

### 4.4. Carthamus tinctorius L.

*Carthamus tinctorius L.*, commonly known as safflower in China, was used to promote blood circulation and remove blood stasis, which was recorded as early as in the *Kaibao Bencao* [70]. The chemical constituents of safflower are plentiful and include flavonoids (e.g., quinochalcone C-glycosides), alkaloids, phenolic acids, and fatty acids [71]. Modern pharmacological experiments have demonstrated that safflower has wide-reaching biological activities, including anticoagulation, antioxidation, antihypoxic, anti-inflammation, and protection of cardiovascular and cerebrovascular [72, 73]. Early literature has reported that safflower injection has significant antioxidant activity outside, and its chemical basis may be polyphenols [74]. Both the medium- and high-dose groups of safflower extract can significantly increase the activities of SOD, GSH-Px, and CAT in brain tissue and reduce the content of MDA in acute cerebral ischemic injury in mice [75]. Safflower yellow is the main active ingredient isolated from safflower, including hydroxysafflor yellow A (HSYA) and safflower yellow B (SYB), which are widely used to treat cerebrovascular diseases [76]. It is reported that safflower yellow has obvious protective effects on rats with cerebral I/R injury by decreasing the levels of MDA and NO and increasing the activity of SOD in brain tissue [77]. SYB is a yellow amorphous water-soluble powder and has demonstrated protective effects in neuronal injury models induced by oxidative stress [78]. Wang et al. studied that the antioxidant effects of SYB were driven by an AK046177/miR-134/CREB-dependent mechanism that inhibited this pathway [23]. SYB attenuated the effects of AK046177, inhibited miR-134 expression, and promoted CREB activation, which in turn promoted Nrf2 expression and then increased antioxidant capacities, improved cell respiration, and reduced apoptosis [23]. Wei et al. showed that HSYA might oppose cerebral I/R injury of MCAO rats through attenuating the elevation of the MDA level and decreasing SOD activity in the ipsilateral hemisphere and serum [79]. In an *in vitro* assay, HSYA was shown to block OGD/R-induced PC12 cell apoptosis through the suppression of intracellular oxidative stress [80]. And another study reported that the synergistic protective effect of HSYA and AST IV could increase the activity of SOD, CAT, and GSH-Px; decrease MDA and ROS; and upregulate the expression of Nrf2 in cerebral I/R injury rats [81].

### 4.5. Angelica sinensis

The dried root of *Angelica sinensis* (Oliv.) Diels, commonly known as Danggui (in Chinese), has been used over thousands of years as well-known Chinese medicines [82]. It has a therapeutic effect on diseases by promoting blood circulation, regulating menstruation, and relieving pain.

With the modernization of TCM, the main components of Danggui have been identified including polysaccharides, organic acids, volatile oils, and flavonoids, as well as vitamins, amino acids, etc. [82, 83]. And modern pharmacological experiments have demonstrated that Danggui could promise neuroprotective effects against ischemic-induced injury by antioxidative stress, antiapoptotic, and anti-inflammatory [82].

The *Angelica sinensis* polysaccharide (ASP) is one of the main extracts from the root of *Angelica sinensis*. One literature reported that pretreatment with ASPs 100 or 300 mg/kg has protective effects for cerebral I/R injury rabbits through increasing the activities of SOD, CAT, GSH-Px, and GR and reducing the production of MDA and NO [84]. In addition, another literature indicated that ASP not only protected PC12 neuronal cells from H_2_O_2_-induced oxidative and apoptotic injury but also promoted the recovery of MCAO rats from cerebral I/R injury, suggesting that ASP has potential as a neuroprotective agent [85]. It is reported that pretreatment with ASPs 30 or 60 mg/kg could increase the activity of SOD and GSH-Px and decrease MDA in MCAO rats [86].

### 4.6. Others

The consumption of polyphenol-rich foods has been related to a lower risk of cardiovascular events (cardiovascular mortality, myocardial infarction, and stroke) and cardiovascular risk factors [87]. Curcumin, a polyphenol abundant in the rhizome of the turmeric plant (Curcuma longa), has shown promising neuroprotective effects in animal models of neurodegenerative diseases [88]. Curcumin could prevent mitochondrial dysfunction as it acts by enhancing the action of enzymes of the antioxidant defense system SOD, CAT, and GSH [89]. Besides, in the rat model of ischemia, Mucuna pruriens extract demonstrated antioxidant capacity against brain damage, which indicated the therapeutic potential of this plant in ischemia [90].

## 5. Conclusion and Prospect

Because the research on ischemic stroke is still in the cognitive stage, most of the mechanisms of action are still unclear, so the diagnosis and treatment methods are still flawed. Therefore, further in-depth study of the mechanism of ischemic stroke is of great help in understanding and treating the disease. By arranging the literature, it was found that TCM has a variety of biological activities and antioxidant capacity and can protect against ischemic stroke by regulating oxidative stress, which indicates that TCM has the potential to protect the body from ischemic stroke by antioxidative stress (Table 1). Through the analysis of the existing literature, we found that the antioxidant effect of TCM is the result of multifaceted and multimechanism. TCMs can directly enhance the activity of endogenous antioxidant enzymes (such as SOD, GSH-Px, and CAT) to defend against oxidative stress. In addition, TCMs can modulate signaling pathways related to ROS, such as the Nrf2 pathway (Table 1). And TCMs also can directly reduce the oxidative damage of cellular macromolecules (such as lipids, proteins, and DNA).

Collectively, we first discuss the redox signaling and oxidative stress pathways in ischemic stroke and propose that inhibiting of oxidative stress is a potential target for the treatment and prevention of ischemic stroke. Then, we summarize recent research data and discuss the action mechanism of Chinese herbal medicine and its active ingredients in preventing ischemic stroke by modulating redox signaling and oxidative stress pathways. Due to its antioxidant ingredients, TCM treatment has particular advantages in the treatment of ischemic stroke. But one of the biggest challenges in modernizing TCM is the lack of robust clinical trials. TCM with ischemic stroke treatment effects contain complex and diverse types of active ingredients. Although current studies have found that the active ingredients contained in TCM can play a protective role by regulating oxidative stress to deal with cerebral I/R damage, the mechanism of action is not sufficiently studied, the research scope is relatively limited, and the research indicators are relatively single. It is unclear how these active ingredients work on this target. Thus, aiming at this target, researchers should actively design a plan, through real preclinical research and scientific clinical trials, to explore whether TCM antioxidant treatment can become a breakthrough point in the treatment of ischemic stroke and provide therapeutic strategies and theoretical basis for the clinical treatment of ischemic stroke. By adding more experimental and clinical data to increase the theoretical support of TCM against oxidative stress, we further optimize the active ingredients, dosage, administration time, and administration method of TCM. This will help to facilitate the natural anti-ischemic stroke medicine discovery and development and its bench-to-bedside transformation. And this also will help to apply these TCMs more safely and rationally to avoid adverse events, improve the quality of life of more ischemic stroke patients, and have important application value in clinical practice.

## Figures and Tables

**Figure 1:** The antioxidative systems related to ischemic stroke.

**Table 1:** Mechanisms of TCM and its active ingredients to improve oxidative stress.

TCM	Ingredient	Subjects in study	Impact on ROS-related targets	Refs.
*Ligusticum chuanxiong*	Tetramethylpyrazine	SD rats	↑Nrf2, ↑HO-1	[47]
	Volatile oil	SD rats	↑SOD, ↑GSH-Px, ↓MDA	[48]
*Astragalus membranaceus*	Astragaloside	SD rats	↑SOD, ↓LDH, ↓NOS, ↓MDA, ↓NO	[56]
	Astragaloside IV	SD rats/SH-5Y5Y cells	↓ROS, ↑Nrf2	[57]
	Astragaloside IV-tetramethylpyrazine	SD rats	↓MDA, ↓iNOS, ↑SOD,	[58]
	*Astragalus polysaccharides*	SD rats	↑SOD, ↓NOS, ↓MDA, ↓NO, ↓LDH	[59]
	Calycosin-7-O-*Β*-D-glucoside	HT22 cells	↓LDH, ↓MDA, ↓ROS, ↑SOD	[61]
*Radix Salvia Miltiorrhizae*	Salvianolic acid B	Mice	↓MDA, ↑SOD, ↓NOS, ↑T-AOC	[66]
	Salvianolic acid B	SD rats	↑SOD, ↑CAT, ↑GSH-Px, ↓MDA, ↓LDH, ↓NOS	[67]
	Danshen polysaccharide	Wistar rats	↓MDA, ↓ROS, ↑SOD, ↑CAT, ↑GSH-Px,	[68]
	Tanshinone IIA	*Nrf2* knockout mice	↑Nrf2, ↓8-OHdG, ↓MDA, ↑SOD, ↑CAT, ↑GSH-Px, ↑T-AOC	[69]
*Carthamus tinctorius* L.	Safflower extract	ICR mice	↑SOD, ↑GSH-Px, ↑CAT, ↓MDA	[75]
	Safflower yellow pigment	SD rats	↑SOD, ↓NO, ↓MDA	[77]
	SYB	PC12 cells	↑SOD, ↑GSH-Px, ↓MDA, ↓LDH	[78]
	SYB	SD rats/primary cortical cells	↑Nrf2, ↑SOD, ↓MDA, ↑GSH-Px, ↓NADPH, ↓NOX, ↓ROS	[23]
	HSYA	SD rats	↑SOD, ↑T-AOC, ↓MDA	[79]
	HSYA	PC12 cells	↑SOD, ↓MDA	[80]
*Angelica sinensis*	*Angelica sinensis* polysaccharides	Rabbits	↑SOD, ↓MDA, ↑CAT, ↑GSH-Px, ↑GSH, ↑GR, ↓NO	[84]
	*Angelica sinensis* polysaccharides	PC12 cells	↑SOD, ↑GSH-Px, ↓MDA	[85]
	*Angelica sinensis* polysaccharides	Wistar rats	↑SOD, ↑GSH-Px, ↓MDA	[86]
